# Toward characterization and definition of fibromyalgia severity

**DOI:** 10.1186/1471-2474-11-66

**Published:** 2010-04-08

**Authors:** Stuart Silverman, Alesia Sadosky, Chris Evans, Yating Yeh, Jose Ma J Alvir, Gergana Zlateva

**Affiliations:** 1 Cedars-Sinai Medical Center, Los Angeles, CA, USA; 2 Global Outcomes Research, Pfizer Inc., New York, NY, USA; 3 Mapi Values, Boston, MA, USA

## Abstract

**Background:**

There are no standard criteria for defining or assessing severity of fibromyalgia (FM) as a condition as fibromyalgia is associated with multiple symptom domains. The objective of this study was to evaluate whether patient self-reported severity of FM is associated with severity of pain and sleep interference and the presence of core co-morbidities.

**Methods:**

We recruited individuals ≥ 18 years of age with a clinician-confirmed diagnosis of FM ≥ 3 months and a current pain rating >2 on a 0-10 numeric rating scale (NRS). Patients completed a questionnaire by mail in which they self-rated their FM severity (very mild, mild, moderate, and severe), their current pain severity and extent of sleep interference (NRS; mild, 0-3; moderate, 4-6, severe, 7-10), and provided information (yes/no) on the presence of core comorbidities (symptoms of depression, anxiety, sleep problems, back pain, neck pain) and medication use for FM. The core symptoms of FM were stratified to assist with patient characterization. Analysis of variance (ANOVA) was used to explore the relationship between self-reported FM severity and continuous variables (pain severity and sleep interference), and Mantel-Haenszel chi-square analysis was used to evaluate the trend in the proportions of patients reporting use of medications and core symptoms of FM by severity of FM. To complement patient-reported FM severity and to understand physicians' perspectives, a survey was performed among 28 physician specialists (rheumatology, neurology, anesthesiology/pain management, family practice, internal medicine, and psychiatry) to determine what they assessed when evaluating FM severity in clinical practice.

**Results:**

The population (N = 129) of FM patients was predominantly female (89.1%), with a mean age of 49.4 ± 11.0 years, and 81.4% reported duration ≥ 2 years. Self-reported FM severity was moderate/severe in 86.0% of patients; mean current pain score was 6.40 ± 2.19 (moderate), and mean sleep interference score was 7.28 ± 2.23 (severe). Greater FM severity was significantly associated with higher levels of current pain and sleep interference (p < 0.0001), the proportion of patients reporting FM medication use (p = 0.0001), and the presence of core comorbidities (p < 0.05). Pain, functional disability, and fatigue severity were ranked as the top three criteria by the highest proportion of physicians when evaluating FM severity.

**Conclusion:**

With higher self-reported FM severity, patients have greater pain and sleep interference as well as increased frequency of core comorbidities. Further investigation into understanding FM severity is warranted.

## Background

Fibromyalgia (FM) is a disorder of unknown etiology that is generally diagnosed according to the American College of Rheumatology (ACR) criteria, which include chronic, widespread pain for at least 3 months, and the presence of 11 out of 18 tender points [1]. Prevalence estimates for the United States suggest that approximately 5 million individuals have this condition, with a higher prevalence among women (3.4%) than men (0.5%) [2]. Although chronic widespread pain is the hallmark of FM, core symptoms of FM also include sleep disturbance, fatigue, mood disorders, and localized pain (headache, back and/or neck pain). These core symptoms are included among the domains that have been identified and recognized by OMERACT (Outcomes Measures in Rheumatology) as important for assessment in FM [3].

FM has a substantial negative impact on quality of life, resulting in health status that is poorer than other chronic pain conditions such as rheumatoid arthritis and osteoarthritis [4-7]. The burden imposed by core FM symptoms translates into limitations of productivity, personal and family life, as well as a reduced ability to complete simple activities of daily living [6,8].

This multidimensional nature of FM has made it difficult to define and assess the severity of FM as a condition. The indeterminate etiology and lack of specific disease markers exacerbate the problem of assessing FM severity. While several studies investigated the potential use of biologic markers for FM (e.g. cytokines, antipolymer antibodies), correlation of these markers with symptoms was equivocal at best [9-12], rendering them ineffective as indicators of severity. Similarly, although tender points and a total myalgic score have been evaluated as measures of severity [13,14], they demonstrate inherent variability over time [13], show little correlation with other outcome measures, and importantly, neither is of clinical relevance to patients. A recent comprehensive review of potential FM biomarkers highlighted the lack of appropriate evaluation of objective biomarkers of FM, although limited data from a longitudinal study suggested that the results obtained during experimental pain testing were associated with clinical status improvements [15]. However, it should be noted that in addition to sensitivity to change with clinical improvement, biomarkers need to demonstrate change with worsening disease if they are to be considered indicators of disease severity.

The ability to evaluate and measure the severity of FM as a condition is likely to provide several benefits including identification of treatment responders in clinical trials and clinical practice. Characterization of severity levels may also be used as a marker for disease progression. Treatment approaches may be specifically targeted to patients at different levels of severity, with the potential for determining if early treatment may slow or prevent disease progression. There have been few published studies on severity or progression of FM as a disease state, and what little has been reported about the natural history of FM is inconsistent. Although a longitudinal study by Wolfe et al. reported no change in the severity of specific symptoms over time [16], a review of the few published studies suggested no clear pattern of progression or remission [17].

Chronic pain is the symptom of FM that is of primary importance to patients and clinicians and is routinely evaluated as an endpoint in clinical trials and clinical practice. Although pain can be quantitatively evaluated from the patient's perspective, it may not be an adequate surrogate of disease severity, since it may display intrapatient variability in intensity which does not necessarily correlate with the presence or severity of other FM symptoms. A patient-reported instrument frequently used to assess FM is the Fibromyalgia Impact Questionnaire (FIQ) [18]. Although the FIQ is sensitive to treatment effects [19], it evaluates the impact of FM on various activities which may be related to, but does not actually measure, disease severity. Furthermore, the FIQ appears to have low sensitivity to clinical worsening [19], and it is unlikely to be an accurate indicator of disease severity.

In trying to develop a model of FM severity, Goldenberg et al. [20] evaluated 15 potential explanatory factors in a regression analysis. Several of the items evaluated, including pain and psychological distress, may relate to severity as contributory factors. However, others such as employment status, pending litigation, and education level, may be associated with severity in terms of impact but are not adequate for providing a definition of FM severity as a disease state.

A study by Giesecke et al. [21] used cluster analysis to classify patients with FM into subgroups based on levels of mood, catastrophizing, perceived control over pain, and tenderness. While this attempt at categorization demonstrated an ability to place patients into one of three groups (moderate mood, catastrophizing and perceived pain control with low tenderness; elevated mood assessment, catastrophizing, and tenderness with low control over pain; and normal mood and catastrophizing with high pain control but extreme tenderness), these results were not placed in the overall context of disease severity.

The purpose of the current study was to initially characterize FM severity from the perspective of individuals with FM and to determine if patients' perception of FM severity is more than simply their pain. We utilized data from a larger FM patient study to conduct a post-hoc exploratory analysis of symptom severity. Data were collected on several self-reported parameters including patient-rated disease severity and the presence of core comorbid conditions, we report here the preliminary evaluation of whether patient self-reported severity of FM is associated with corresponding severity of pain and sleep interference and the presence of core co-morbidities. This patient perspective is also complemented with the results of a small physician survey designed to understand the physicians' perspective by capturing information on what characteristics the physicians use to assess FM severity in their daily clinical practice.

## Methods

Patients were recruited through newspapers, support groups, and the internet as part of a larger patient reported outcome study conducted in the US to Patients were compensated for participation. For inclusion, patients had to be ≥ 18 years of age with a clinician-confirmed diagnosis of FM ≥ 3 months (based on a review of each patient's medical record). Clinicians could be either specialists or general practitioners, and was likely dependent upon the duration of FM since diagnosis. A current pain rating >2 on a 0-10 numeric rating scale (NRS) from the modified Brief Pain Inventory short form (mBPI-sf) [22] was also required for inclusion, as was an ability to understand and read English. The presence of rheumatoid arthritis, systemic lupus erythematosus, or any other chronic pain condition that would confound the ability to distinguish the chronic pain from pain related to fibromyalgia was reason for exclusion.

Responses to questions were obtained using a mail-in mail-back questionnaire. Subjects interested in participating were mailed the questionnaires in packets containing written instructions on questionnaire completion and guidance for frequently asked questions. In addition, a researcher from Mapi Values contacted the subjects to review the materials and ask if they had questions on completing the forms. Subjects were also provided a toll free number to call for study-related questions. All study screening materials, informed consent, demographic forms, protocol and other study documents were submitted and approved by the Copernicus Group Institutional Revew Board (IRB), an independent IRB (approval granted on May 10^th ^2007).

Patients self-rated their FM severity (very mild, mild, moderate, and severe) and provided an evaluation of their current pain severity using the 11-point NRS. Sleep interference was assessed using the sleep interference item from the mBPI-sf, a 0-10 NRS that asks "How, during the past 24 hours, pain due to your fibromyalgia has interfered with your sleep?" Cutoff scores of 0-3, 4-6, and 7-10 were used to characterize mild, moderate, and severe NRS ratings, respectively. These cutpoints were used since they have been previously identified as being optimal for classifying pain in a neuropathic pain condition (painful diabetic peripheral neuropathy) [23]. Additionally, the presence of comorbidities was reported by patients (yes/no for symptoms of depression, anxiety, sleep problems, back pain, neck pain) as was medication use for FM (yes/no).

Patient responses and scores were stratified by self-reported FM severity. Analysis of variance (ANOVA) was used to explore the relationship between self reported FM severity and the continuous variables of pain severity and sleep interference scores, and Mantel-Haenszel chi-square analysis was used to test for trend in the proportions of patients reporting use of medications and core symptoms of FM by severity of FM.

To complement the characterization of FM severity as reported by patients, the results of a small, separate physician survey are presented that aimed to explore FM severity from the perspective of the clinician. This survey was performed among 28 physicians considered experts in their respective specialties (rheumatology, neurology, anesthesiology/pain management, family practice, internal medicine, and psychiatry). The physicians were asked to respond to the question "When you assess the severity of fibromyalgia *as a condition *in your patients, what are the top 5 items (specific symptoms, specific physical findings, specific abnormal lab findings, etc.) that influence your decision-making?" Descriptive analysis was used to evaluate the rankings by proportion of physicians reporting each criterion.

## Results

### Patient-reported severity

A total of 129 patients were enrolled in the study, and the demographics (Table 1) show that this population was predominantly female (89.1%), the mean age was 49.4 ± 11.0 years, and almost half the patients (47.3%) were employed at least part time. The majority of patients (81.4%) reported FM (≥ 2 years), and approximately one-quarter of the patients (25.6%) had FM > 10 years.

**Table 1:** Demographic characteristics of the population (N = 129)

Characteristic	Value
Age, y	
Mean ± SD	49.4 ± 11.0
Median	50.0
Range	23.0-78.0
Missing data, n (%)	3 (2.3)
Gender, n (%)	
Female	115 (89.1)
Male	11 (8.5)
Missing data	3 (2.3)
Employment status, n (%)	
Employed full time	38 (29.5)
Employed part time	23 (17.8)
Homemaker	16 (12.4)
Retired	11 (8.5)
Unemployed	11 (8.5)
Other	25 (19.4)
Missing data	5 (3.9)
Duration of fibromyalgia, n (%)	
3 months-1 year	20 (15.6)
2-5 years	44 (34.1)
6-10 years	28 (21.7)
> 10 years	33 (25.6)
Missing data	4 (3.1)
Current pain severity^a^	
Mean ± SD	6.40 ± 2.19
Range	0.0 - 10.0
Median	7.0
Missing data, n (%)	13 (10.1)

^a ^0-10 numerical rating scale from the short form Modified Brief Pain Inventory

While 111 patients (86.0%) reported their FM severity as being of at least moderate intensity (45.7% moderate and 40.3% severe), 3 patients (2.3%) and 12 patients (9.3%) reported very mild and mild severity, respectively. Due to the low number of patients in the very mild category, this category was collapsed into the mild category representing 15 patients (11.6%). Data were missing for 3 patients (2.3%). The mean NRS scores from the mBPI-sf suggested current pain of moderate severity (6.40 ± 2.19), and pain-related sleep interference that was severe (7.28 ± 2.23). As shown in Figures 1A and 1B for both of these outcomes, with greater self-reported FM severity, there was a corresponding increase in pain severity and sleep interference. ANOVA analysis suggested that this higher FM severity was significantly associated with the increase in current pain (*F *[2, 113] = 21.10, *p *<0.0001 and sleep interference (*F *[2, 113] = 15.4, *p *<0.0001). Sleep interference scores were higher (i.e. greater severity) than pain scores at all levels of FM severity.

**Figure 1:** **Relationship between self-reported fibromyalgia severity and current pain (A) and pain-related sleep interference (B)**. Values represent mean scores (± standard deviation as shown by the vertical bars) from the short form of the modified Brief Pain Inventory. P values are for the overall association between fibromyalgia severity and levels of current pain and pain-related sleep interference using ANOVA.

Similarly, at higher levels of self-reported FM severity, there was a corresponding increase in the proportion of patients who used medications for their FM and who reported core comorbidities including sleep problems, depression and anxiety, and back and neck pain (Table 2). Among patients with severe FM, 90% had sleep problems and 84% were using medications for FM. Even among patients with mild FM, sleep problems were reported by 40% of the patients, and prescription medications for FM were used by approximately one quarter (26.7%) of the patients. For nearly all levels of FM severity, the proportion of patients reporting symptoms of depression was similar to the proportion reporting symptoms of anxiety. The exception was for mild FM, of which a higher proportion of patients (20.0%) reported symptoms of anxiety relative to depression (6.7%). Mantel-Haenszel chi-square tests suggested that the trends observed with increasing self-reported severity were significant for medication use and all core comorbidities (Table 2).

**Table 2:** Relationship between self-reported fibromyalgia severity and proportion of patients reporting use of medications and core symptoms of fibromyalgia (FM).

**Binary Variable**	**Self-reported FM severity** **(percent of patients)**			**Mantel-Haenszel Χ^2^** **(P value)**
	**Mild**	**Moderate**	**Severe**	
		
Medications for FM	26.7	65.5	84.0	16.54 (< 0.0001)
Sleep problems	40.0	72.9	90.4	15.99 (< 0.0001)
Symptoms of depression	6.7	52.5	65.4	13.14 (< 0.001)
Symptoms of anxiety	20.0	52.5	61.5	6.56 (< 0.05)
Back pain	46.7	72.9	82.7	6.90 (< 0.01)
Neck pain	26.7	72.9	71.2	5.52 (< 0.05)

Mantel-Haenszel chi-square tests for trend (d.f. = 1) of the proportions of patients reporting use of medications and core symptoms of fibromyalgia by severity of fibromyalgia.

FM severity was also significantly associated with duration of FM since initial diagnosis (Figure 2; Chi-square = 27.22; df = 6; p = 0.0001). The majority of patients who reported mild FM (60%) had been diagnosed with FM during the previous year, and conversely, 94% of patients with FM duration ≥ 2 years since diagnosis reported moderate to severe FM.

**Figure 2:** **Relationship between duration of fibromyalgia and patient self-reported fibromyalgia severity**. The percentages reflect the proportion of patients with the indicated duration of fibromyalgia who were at each self-reported severity level (e.g. of patients with fibromyalgia < 1 year, 45% reported mild disease). Chi-square = 27.22, df = 6; p = 0.0001.

### Physician reported severity

When asked to provide a ranked list of the top 5 items that contribute to decision-making when evaluating patients with FM, physicians listed a variety of criteria that they use for assessing FM severity. Table 3 presents the results of the survey by arranging the items according to the highest proportion of physicians who gave a designated rank to a specific symptom. Pain, functional disability, and fatigue severity were ranked as the top three criteria by the highest proportion of physicians. The greatest concordance was for pain, which was ranked as the top criterion by 17 of the 28 physicians (61%), although physicians also cited several other factors considered as primary criteria, including the Fibromyalgia Impact Questionnaire score, functional disability, and tender points. While sleep disruption was not included in the top three criteria, it was nevertheless used as a criterion of FM severity by 43% of physicians, as were the presence of comorbidities (32%) and duration of symptoms (18%).

**Table 3:** Ranked criteria reported by physicians for assessing fibromyalgia severity (N = 28) based on the open-ended question "When you assess the severity of fibromyalgia *as a condition *in your patients, what are the top 5 items (specific symptoms, specific physical findings, specific abnormal lab findings, etc.) that influence your decision-making?"

Ranked criteria, n (%) of responses				
#1	#2	#3	#4	#5
Pain*, 17 (60.7)	Functional disability, 6 (21.4)	Fatigue, 4 (14.3)	Functional disability, 4 (14.3)	Fatigue severity, 3 (10.7)
FIQ, 3 (10.7)	Pain, 4 (14.3)	Functional disability, 3 (10.7)	Presence of comorbidities, 4 (14.3)	Duration of symptoms, 1 (3.6)
Functional disability, 2 (7.1)	Sleep disruption, 4 (14.3)	Sleep disruption, 3 (10.7)	Sleep disruption, 3 (10.7)	Pain, 1 (3.6)
Tender points, 2 (7.1)	Duration of symptoms, 3 (10.7)	Presence of comorbidities, 3 (10.7)	Fatigue severity, 2 (7.1)	Sleep disruption, 1 (3.6)
Fatigue, 1 (3.6)	Tender points, 2 (7.1)	Pain, 2 (7.1)	Pain, 1 (3.6)	Global assessment,1 (3.6)
QoL, 1 (3.6)	Presence of comorbidities, 2 (7.1)	Tender points, 2 (7.1)	QoL, 1 (3.6)	Tender points, 1 (3.6)
Sleep disruption, 1 (3.6)	Fatigue, 1 (3.6)	QoL, 1 (3.6)	Other, 5 (17.9)	Number of medications, 1 (3.6)
Clinical history, 1 (3.6)	FIQ, 1 (3.6)	Duration of symptoms, 1 (3.6)	None listed, 7 (25.0)	Other, 7 (25.0)
	HAQ, 1 (3.6)	Global assessment, 1 (3.6)		None listed, 12 (42.9)
	Other^†^, 2 (6.9)	Number of medications, 1 (3.6)		
	None listed, 1 (3.6)	Other, 4 (14.3		

FIQ, Fibromyalgia Impact Questionnaire; QoL, Quality of life; HAQ, Health Assessment Questionnaire. *Pain includes intensity and/or quality characteristics. ^†^"Other" category includes laboratory abnormalities, cognitive/behavioral status, psychological impact, work status

Columns are ordered by decreasing rank, rows are ordered by the proportion of physicians designating a particular numerical rank for the specific symptom.

## Discussion

This study suggests that the association of FM severity with symptoms that have been identified as being of clinical importance by patients and physicians [3], and are considered by OMERACT to be among the core FM symptoms for evaluation [3,24], may be useful for the characterization and assessment of the severity of FM as a condition. In particular, with higher self-reported FM severity, i.e. from mild to moderate to severe, an associated increase was observed in pain, sleep disturbance, and depressive symptoms, as well as the use of medications for FM and the presence of comorbid conditions including back and neck pain. Therefore, these characteristics may contribute to the patient's overall perception of disease severity.

Determining a definition of FM severity could be helpful for disease management. A definition based on the patient's perspective may be especially useful, since in the absence of objective disease biomarkers it relies on readily available information of clinical relevance to the patient that can be used by physicians for patient classification and management. The only other study that attempted to develop a severity model also used a patient-reported outcome, global VAS, as the anchor for FM severity [20]. While the current study did not use a validated measure, the anchor for FM severity was a question specifically addressing FM rather than a global assessment.

The use of patient self-report is increasingly being accepted and applied as a method to evaluate disease states and management strategies in clinical trials, especially for chronic pain conditions [25]. This has been true for the rheumatic diseases including FM, for which most of the core domains considered by OMERACT as being essential for evaluation, are patient-centric [3,24]. The top five of these domains include pain, fatigue, patient global, sleep, and multidimensional function. These domains are generally the same as those identified as being important by patients, i.e. pain or physical discomfort, aching joints or pain, lack of energy or fatigue, effects on sleep, and problems with attention or concentration [3,24]. Patients may have a better sense of their condition than can be obtained using objective clinical criteria, and at least in some rheumatic conditions, patient-centered outcomes may also discriminate between placebo and active treatment as well as or better than objective clinical measures [26-28].

While two factors identified in this exploratory analysis, i.e. pain and depression, were previously identified by Goldenberg et al. [20] as having a potential relationship with FM severity, the results reported here also suggest that overall, patients with longer FM duration tended to report greater FM severity. However, it should be noted that there was a small increase in the proportion of patients reporting mild severity among the patients with FM duration > 10 years relative to those having a shorter duration. Although the reason for this increase was not explored, it could potentially be due to adaptation or a greater ability to cope with a chronic condition among some patients. This is consistent with what was reported by Kennedy et al. [29] in one of the few long-term (10-year) follow-up of patients with fibromyalgia; at 10 years, despite the presence of symptoms that showed little change from the initial survey and continued use of medication, a substantial proportion of patients reported that they felt better in terms of FMS symptoms.

The observed relationship between FM severity and duration is in contrast to Goldenberg et al. [20] who reported that there was no relationship between these variables. Their observation may potentially result from use of a global assessment rather than a more specific FM assessment [20]. Similarly, the results reported here diverge from a previous study which reported that symptom severity does not change over time [16]. However, that study used more compressed assessment scales for sleep disturbance and pain (0-3 visual analogue scales) than the current study (0-10 NRS) and did not stratify patients by FM duration. If such an association between duration and severity can be confirmed, it may provide an opportunity to identify patients early in the disease continuum and eventually modify or delay disease progression through the use of pharmacological and/or non-pharmacological interventions.

The observation that the NRS scores for sleep disturbance were higher than NRS pain scores across all levels of FM severity appears to be consistent with a recent analysis showing that sleep problems were predictive of pain [30], although it is unlikely that the relationship between sleep and pain is unidirectional. However, the data do suggest that these two variables may be central, although not exclusive, components for defining severity of FM, and that management of both pain and sleep problems are integral to the treatment of FM.

In contrast to the patient survey, which was closed-ended and elicited severity information based on specific symptoms and comorbidities, the physician survey was open-ended. This physician survey demonstrated that, consistent with the absence of an adequate definition of FM severity, there was a general lack of consensus regarding criteria that physicians use as an indicator of FM severity. That pain was the most frequently used criterion of severity was not surprising considering that pain is often the primary complaint of patients with FM. However, despite being ranked first as an indicator of severity, only 61% of the physicians considered pain the primary criterion. There was little concordance on the use of other criteria, including several of the factors that demonstrated a relationship with higher levels of self-reported FM severity, i.e. sleep interference and the presence of comorbidities, which were identified by only 43% and 32% of physicians, respectively. The small sample size (N = 28) may have contributed to this lack of concordance.

Although functional disability was ranked second and fatigue was ranked third, these criteria were used overall by 54% and 39% of physicians, respectively. These particular criteria, although identified by physicians, were not assessed in patients as part of the patient survey, and may be considered a limitation of the study, especially since fatigue is a frequent complaint among patients with FM [31]. Indeed, while the patient and physician surveys provide complementary information regarding perceptions of FM severity, the different manner in which the surveys were performed precludes comparison of these surveys, since patients were asked to rate severity but were not asked to rank symptoms.

Since physicians identified and ranked criteria in response to a question ("When you assess the severity of fibromyalgia *as a condition *in your patients, what are the top 5 items [specific symptoms, specific physical findings, specific abnormal lab findings, etc.] that influence your decision-making?"), physicians were not specifically queried as to how these assessments are made. It should be noted that objective clinical assessment using tender points was cited by only 18% of the physicians, and that nearly all the other criteria were patient-centric. The variety of criteria that these physicians, who routinely treat FM patients, reported using and the lack of concordance on their use, reinforces the need to define what constitutes an adequate measure of FM severity. Being able to define and measure FM severity may have practical benefits in terms of understanding disease progression and evaluating treatment approaches for their potential ability to slow progression. The ability to slow progression is likely to have a broader clinical and economic impact by reducing health resource utilization and associated costs.

This was an exploratory, post-hoc analysis and is subject to several limitations. As part of the eligibility criteria, participants were required to have a minimum level of pain, i.e. a current pain rating of at least 2 on a 0-10 NRS. In addition to the small sample size, this inclusion criterion may have selected against patients who would likely have self-reported very mild or mild disease. In fact the proportion of patients in this study who reported these levels of FM severity was small (11.6%), and these levels were mainly associated with FM duration ≤ 1 year, for which the proportion of patients was also correspondingly small (15.9%). Because of these low proportions, the current analysis may have had limited power to evaluate correlations at this end of the severity spectrum.

Furthermore, while the assessments were specific for the variables measured, only single items were used for most of the variables, potentially restricting interpretation of our findings. Additionally, for those outcomes evaluated based on an NRS score (i.e. pain and sleep interference), there is no validation of cutoff scores designating severity levels. Therefore, it cannot be definitively stated that a particular self-reported FM severity level correlated with a similar severity of pain or sleep interference. However, extrapolation of pain ranges for the mBPI-sf (mild 0-3, moderate 4-6, severe 7-10) that were validated for a neuropathic pain condition, diabetic peripheral neuropathy [23], suggests that these outcomes were of at least moderate intensity even among FM patients who self-reported mild FM.

The fact that patients were compensated for participation may have introduced additional bias, since it is not known what effect the use of compensation may have had on the selection of patients. Consequently, the results reported here may not be generalizable to the overall FM population. The small number of patients, although representative of various regions of the US, may also contribute to the lack of generalizability. There were a disproportionate number of female participants, with the implication that gender bias may have skewed the data, since gender differences may be operative in the perception and report of pain as well as in the determinants that contribute to self-rated health status [32-34]. However, the sex ratio in this study is not only reflective of FM in clinical practice, but complements the reporting that few gender differences exist in the severity or range of symptoms for FM including pain severity, physical function, and psychological factors [35].

## Conclusions

This study explored the patient and physician perspective of FM severity. With greater patient reported FM severity, there was an increase in other patient reported variables including pain and sleep interference, presence of comorbid conditions and use of medications for FM. This study also suggests that physicians use different domains to rank FM severity. Both these findings need to be validated in further studies. When evaluating severity of FM, physicians should consider the patient perspective.

## Competing interests

Drs. Alvir, Sadosky, and Zlateva are all employees of Pfizer, Inc. Drs. Evans and Yeh are employees of Mapi Values Inc. and received financial support for this project. Dr Silverman is a consultant to Pfizer and Lilly. Dr. Silverman did not receive financial support for this project.

## Authors' contributions

CE and YY designed and initiated the study, and participated in the interpretation of results and manuscript development. SS participated in the interpretation of results and manuscript development. JMJA and YY performed the statistical analyses for the project. AS and GL participated in the analysis and discussion of results, and contributed to manuscript development. All authors read and approved the final manuscript.

## Pre-publication history

The pre-publication history for this paper can be accessed here:

http://www.biomedcentral.com/1471-2474/11/66/prepub
